RETRACTED

# *Mangifera indica* Extracts as Novel PKM2 Inhibitors for Treatment of Triple Negative Breast Cancer

**DOI:** 10.1155/2021/5514669

**Published:** 2021-05-26

**Authors:** Azhar Rasul, Ammara Riaz, Wei Wei, Iqra Sarfraz, Mudassir Hassan, Jiang Li, Faryal Asif, Şevki Adem, Shazia Anwer Bukhari, Muhammad Asrar, Xiaomeng Li

**Affiliations:** ^1^The Key Laboratory of Molecular Epigenetics of MOE, Institute of Genetics and Cytology, Northeast Normal University (NENU), Changchun, China; ^2^Cell and Molecular Biology Lab, Department of Zoology, Faculty of Life Sciences, Government College University Faisalabad, 38000 Faisalabad, Pakistan; ^3^Affiliated Stomatology Hospital of Guangzhou Medical University, Guangzhou, China; ^4^University of Agriculture Faisalabad (UAF), Faisalabad, Pakistan; ^5^Department of Chemistry, Faculty of Science, Cankiri Karatekin University, 18100 Cankırı, Turkey; ^6^Department of Biochemistry, Faculty of Life Sciences, Government College University Faisalabad, 38000 Faisalabad, Pakistan

## Abstract

Pyruvate kinase (PK), a key enzyme that determines glycolytic activity, has been known to support the metabolic phenotype of tumor cells, and specific pyruvate kinase isoform M2 (PKM2) has been reported to fulfill divergent biosynthetic and energetic requirements of cancerous cells. PKM2 is overexpressed in several cancer types and is an emerging drug target for cancer during recent years. Therefore, this study was carried out to identify PKM2 inhibitors from natural products for cancer treatment. Based on the objectives of this study, firstly, plant extract library was established. In order to purify protein for the establishment of enzymatic assay system, pET-28a-HmPKM2 plasmid was transformed to *E. coli* BL21 (DE3) cells for protein expression and purification. After the validation of enzymatic assay system, plant extract library was screened for the identification of inhibitors of PKM2 protein. Out of 51 plant extracts screened, four extracts *Mangifera indica* (leaf, seed, and bark) and *Bombex ceiba* bark extracts were found to be inhibitors of PKM2. In the current study, *M. indica* (leaf, seed, and bark) extracts were further evaluated dose dependently against PKM2. These extracts showed different degrees of concentration-dependent inhibition against PKM2 at 90-360 *μ*g/ml concentrations. We have also investigated the anticancer potential of these extracts against MDA-MB231 cells and generated dose-response curves for the evaluation of IC_50_ values. *M. indica* (bark and seed) extracts significantly halted the growth of MDA-MB231 cells with IC_50_ values of 108 *μ*g/ml and 33 *μ*g/ml, respectively. Literature-based phytochemical analysis of *M. indica* was carried out, and *M. indica*-derived 94 compounds were docked against three binding sites of PKM2 for the identification of PKM2 inhibitors. The results of *in silico* based screening have unveiled various PKM2 modulators; however, further studies are recommended to validate their PKM2 inhibitory potential via *in vitro* biochemical assay. The results of this study provide novel findings for possible mechanism of action of *M. indica* (bark and seed) extracts against TNBC via PKM2 inhibition suggesting that *M. indica* might be of therapeutic interest for the treatment of TNBC.

RETRACTED

## 1. Introduction

Metabolic reprogramming has been reported as an emerging hallmark of cancer in recent years [1]. Reprogrammed tumor metabolism is characterized by enhanced aerobic glycolysis, upregulation of glutaminolysis, and lipid metabolism along with other different bioenergetics pathways which promote cellular growth and survival [2]. Among all these metabolic pathways, glycolysis has been contemplated as the main source of energy for the growing tumor cells [3].

The pyruvate kinase (PK) is a key mediator of glycolytic pathway which codes for four different isoforms in mammalian cells. The oncofetal isoform is the M2 isoform of pyruvate kinase (PKM2) which differs from its M1 isoform by 22 amino acids. PKM1 isoform is expressed in normal cells; however, tumor cells as well as fetal tissues predominantly express the PKM2 isoform [4]. Multiple evidences demonstrate that PKM2 expression support energetic and macromolecular biosynthetic requirements of tumor cells by allowing the accumulation of glycolytic intermediates [5]. PKM2 is overexpressed in numerous kinds of human cancers mainly breast, prostate, lung, colorectal, and hepatocellular carcinoma. Previous studies have also demonstrated that PKM2-mediated glycolysis plays a critical role in tumor development, propagation, survival, and migration of cancer cells; thus, PKM2 inhibition has potential to inhibit growth of cancer cells selectively [6].

Given that PKM2 could serve as an ideal drug target for cancer [7], it is of immense interest to identify its natural inhibitors from natural products (NPs). Through long history of traditional medicinal applications, NPs have been well accepted by oncologists and pharmacologists as a worthwhile database for screening of bioactive extracts and compounds for novel drug discovery [8]. Previous studies have also demonstrated that NPs have promising ability to hit different metabolic targets in cancer cells. Thus, NP-mediated metabolic reprogramming is an emerging trend in the recent years for the development of novel anticancer therapies [9]. Although shikonin has been reported as a potent inhibitor of PKM2 [10], however, poor solubility and toxicity have limited its clinical applications [11]. The investigations on the identification and characterization of PKM2 inhibitors are ongoing, and the discovery of novel, potent, and safer inhibitors with good bioavailability and low toxicity has potential to provide great benefit to cancer patients. Based on this context, the aim of this work was to evaluate the potential of various plant extracts belonging to Pakistani flora against PKM2.

RETRACTED

Based on the aims and objectives of this study, we have screened plant extract library using an *in vitro* enzymatic kinetic assay system for the identification of PKM2 inhibitors. Here, we present biochemical and cell-based evidences suggesting that *Mangifera indica* seed coat and bark extracts target PKM2 and possess anticancer activity against MDA-MB231 cells.

## 2. Materials and Methods

### 2.1. Preparation of Plant Extract Library

Various plants (35) belonging to different families were collected across the Punjab province of Pakistan. The specimens of plants were deposited at Herbarium for identification by Dr. Qasim, Assistant Professor, Department of Botany, GCUF. Plants were washed by water after collection and identification, followed by air drying at a shady place. After drying, the plant matter was subjected to grinding till a coarse powder was obtained. Plant extracts were prepared using Soxhlet apparatus. Methanolic extract was further concentrated using a rotary evaporator at reduced activity and solidified in the freeze drier.

### 2.2. Construction of pET-28a-PKM2 Plasmid

The amplification of coding region of full-length human PKM2 (accession number NM_002654.6) was done from human cells with the following primers: PKM2-Fw: 5′- GAC TCA GAT CTC GAG ATG TCG AAG CCC CAT AGT GAA GC -3′; PKM2-Rev: 5′- CGA CTG CAG AAT TCG CCG CAC AGG AAC AAC AC -3′. Agarose gel electrophoresis was done to fractionate the amplicon. This amplicon was then recovered by using a Qiagen Gel Purification column. Cloning of the coding region of PKM2 was done in expression vector pET28a. Sequence was validated by Sanger sequencing.

### 2.3. Expression and Purification of rPKM2 Protein

Transformation of recombinant plasmid pET-28a-PKM2 was done in the *E. coli* BL21 (DE3) cells. Transformed colony was transferred to 25 ml of LB medium supplemented with a suitable antibiotic, i.e., Kanamycin (50 *μ*g/ml) for incubation. Inoculated culture medium was left for overnight at 37°C. After that, the cultured medium was centrifuged at 6000 rpm for 30 min. 5 ml from this suspension was again inoculated in LB medium (500 ml) with Kanamycin (50 *μ*g/ml). This medium was allowed to grow at room temperature with shaking, till the OD_600nm_ that reached to 0.6. IPTG (0.1 mM) was added and cells were collected by centrifugation after the OD_600nm_ reached to 0.6 and was kept at -20°C for freezing purpose. Followed by freezing, further steps were performed at 4°C. The frozen cell paste was suspended in salt Lysis Buffer which contains the following chemicals: 30 mM NaCl, 50 mM NaH_2_PO_4_, 1M NADP^+^, 1.4 mM *β*-mercaptoethanol, 0.5 mM PMSF, and 10 mM Imidazole. Protease inhibitor cocktail was added as supplementation. Egg white lysozyme was added in the quantity of 0.1 mg/ml, after half an hour. After two hours of incubation for this mixture, 1 h Benzonase treatment was performed. 3 M NaCl stock was added to adjust NaCl to 300 mM, and the lysate was incubated for one hour prior to its centrifugation at 14000 rpm for a time period of 30 min. The clear lysate obtained after centrifugation was subjected to Ni-NTA column which was preequilibrated with Lysis Buffer (10 ml). Lysis Buffer was prepared by adding 300 mM NaCl, 0.5 mM PMSF, 50 mM NaH_2_PO_4_, 1.4 mM *β*-mercaptoethanol, 10 mM Imidazole, and 1M NADP^+^. Maximum binding was ensured for flow-through fraction by reloading it twice. Lysis Buffer (10 ml) and Wash Buffer which comprised of 300 mM NaCl, 50 mM NaH_2_PO_4_, 1M NADP^+^, 20 mM Imidazole, 1.4 mM *β*-mercaptoethanol, and 0.5 mM PMSF was used for washing of Ni-NTA column. Then the recombinant PKM2 protein was exposed to elution buffer 1 (300 mM NaCl, 0.5 mM PMSF, 50 mM NaH_2_PO_4_, 250 mM Imidazole, 1.4 mM b-mercaptoethanol, and 1M NADP^+^) followed by exposure to Elution Buffer 2 (50 mM NaH_2_PO_4_, 300 mM NaCl, 0.5 mM PMSF, 500 mM Imidazole, 1.4 mM b-mercaptoethanol, and 1M NADP^+^). The two elutions were kept separated and treated with 1X PBS, 1M NADP^+^, 0.5 mM PMSF, and 1.4 mM *β*-mercaptoethanol. The final elutions were diluted by addition of glycerol (80%) and stored at -20°C in aliquots [12].

RETRACTED

### 2.4. Establishment of PKM2 Enzymatic Assay System

LDH assay was established in order to investigate the PKM2 inhibitory activity of plant extracts. Plant extracts were dissolved in DMSO to 10 mg/ml, then diluted tenfold with pure water. At 25°C, 200 ng/*μ*l of test extract was incubated for 1 hour in a solution containing 100 mM KCl, 50 mM HEPES, 0.2 mM NADH, 10 mM MgCl_2_, 2 mM ADP, 2 mM phosphoenolpyruvate, and 8 units LDH/ml. With the help of compared change in absorbance at 340 nm, the relative pyruvate kinase activity was calculated.

### 2.5. Cell Culture

Human triple negative breast cancer (TNBC) cells, MDA-MB231, were cultured in DMEM supplemented with FBS (10%) and 100 IU/ml penicillin streptomycin. Cancerous cells were allowed to grow in a CO_2_ incubator at 37°C with the supply of 5% CO_2_ [13].

### 2.6. MTT Cytotoxic Assay

The anticancer activity of plant extracts was assessed by MTT assay. For this purpose, MDA-MB231cells were seeded in 96-well plates. After 12-18 hours, cancerous cells were treated with the various doses of plant extracts for 48 hours. Further, 10 *μ*l of MTT (5 mg/ml) was added and cells were then incubated for 4 hours at 37°C. Then, media was aspirated and 150 *μ*l of DMSO was added. As the last step, absorbance was checked at 490 nm on an ELISA plate reader (Thermo Scientific) [14]. Percentage cell viability was calculated by following formula:

(1) $$\begin{array}{c} \text{Percentage cellular viability}=\frac{\text{Absorbance of treated cells }}{\text{Absorbance of control }}\times 100. \end{array}$$

### 2.7. Docking Studies

The X-ray crystallography structure of the human pyruvate kinase M2 (PKM2) was obtained from the https://www.rcsb.org/structure6V74 [15]. Proteins were imported to a Molegro Virtual Docker [16] and prepared for docking. Water molecules at crystal structure were removed; protein structure errors were checked. The binding regions of 1,6-di-O-phosphono-beta-D-fructofuranose (FBP), amino acids (AA), and oxalate ion/phosphoenolpyruvate (PEP) were determined to docking. Results were reported as MolDock Score. Each docking cavity was defined 16 Å radiuses by selecting the reference ligand center. Binding poses were analyzed by Discovery Studio Visualizer 2021software. The phytochemicals were searched at PubChem database, and their 3D SDF Conformers were downloaded from ZİNC database with InChI Key Codes. They were prepared for docking using UCSF Chimera Software.

## 3. Results

### 3.1. Construction of pET28a-PKM2 Recombinant Plasmid

The recombinant pEGFP-C1-PKM2 plasmid was digested by restriction enzymes, and retrieved DNA fragment was subcloned into a histidine-tagged pET28a vector to generate pET28a-PKM2 recombinant plasmid.  Figure 1(a) shows successfully subcloned PKM2 cDNA into pET28a vector. The double digestion of the recombinant expression plasmid with these restriction enzymes resulted in the generation of two fragments which stand for PKM2 and pET28a backbone, respectively. Sequencing of the plasmid confirmed the correct orientation of insert (PKM2) in the vector (data is not shown).

### 3.2. Expression and Purification of Recombinant PKM2 Protein

Recombinant 6×his-PKM2 plasmid was expressed in BL21-DE3 *E. coli* cells. The recombinant N histidine-tagged protein was purified from *E. coli* cells by using Ni-NTA affinity chromatography. The purified recombinant protein was analyzed on SDS-PAGE. The approximate 58 kDa band on SDS PAGE (Figure 1(b)) represents the successful expression of PKM2 recombinant protein in BL21-DE3 *E. coli* clones.

RETRACTED

### 3.3. Establishment and Validation of PKM2 Enzymatic Assay

Using the purified rPKM2 protein, PKM2 enzymatic assay was established based on the principle that the product of PKM2-catalyzed reaction is converted to lactate by LDH with concomitant conversion of NADH to NAD+ which can be monitored spectrophotometrically. The first enzymatic reaction is coupled with another in order to make PKM2 enzymatic activity easily detectable by monitoring NADH (Figure 1(c)). PKM2 enzymatic activity is spectrophotometrically monitored by measuring the decreased NADH at 340 nm. The reaction conditions were optimized using different concentrations of protein and substrate. The PKM2 enzymatic activity was determined at varying concentrations of PEP (Figure 1(d)). Based on our obtained results, 0.5 mM concentration of substrate was selected for further experimentations.

### 3.4. Screening of Crude Plant Extract Library by *In Vitro* PKM2 Enzymatic Assay

Our established coupled PKM2 enzymatic assay was used to determine the inhibitory potential of 51 extracts from various parts of 35 plants covering over 20 families of the Pakistani flora. In this preliminary screening, the PKM2 inhibiting activities of 51 extracts were investigated at 400 *μ*g/ml, and the obtained results are presented in Table 1. From these screened plant extracts, 7.8% (four plant extracts) were identified as active against PKM2 (>70% inhibition), 9.8% exhibited moderate inhibitory activity against PKM2 (41-70% inhibition), and 82.3% displayed insignificant or low activity (0-40% inhibition).

To find the most potent plant extracts at lower concentrations, we further proceeded with screening of hits at lower concentrations. From these highly active plant extracts, *M. indica* (leaf, bark, and seed coat) extracts were tested dose dependently at varying concentrations (90, 180, and 360 *μ*g/ml) in the reconfirmation assay and dose-response curves were obtained (Figure 2).

The obtained results show that *M. indica* extracts could serve as a starting point for the further identification and isolation of PKM2 inhibitory compounds or development of anticancer functional foods. Thus, these plant extracts were selected for further testing of cytotoxicity against breast cancer.

### 3.5. Evaluation of Cytotoxicity of *M. indica* (Leaf, Bark, and Seed Coat) Extracts and Calculation of IC_50_ Values

In order to evaluate the antiproliferative potential of positive hits obtained after screening of plant extract library against PKM2, MTT assay was performed. *M. indica* leaf, bark, and seed coat extracts were found to be cytotoxic towards MDA-MB231 cells. The dose-response curves were generated to calculate the inhibitory concentrations (IC_50_). *M. indica* (bark, leaf, and seed) extracts have potential to inhibit the growth of MDA-MB231 cells significantly with IC_50_ values of 108 *μ*g/ml, 67 *μ*g/ml, and 33 *μ*g/ml, respectively (Figure 3). Thus, the results of this study provide a novel finding about possible mechanism of action of *M. indica* (bark and seed) extracts against TNBC.

RETRACTED

### 3.6. Identification of PKM2 Inhibitors from *M. indica* via *In Silico* Based Screening

In order to identify the PKM2 inhibitor compounds from *M. indica* extract, phytochemical analysis was done through database searching and a list of *M. indica*-derived compounds reported in literature was prepared. The structures of these phytochemicals (ligands) were retrieved from PubChem database, and screening was performed by molecular docking against PKM2 binding sites. *M. indica*-derived 94 compounds were docked against 3 binding sites of PKM2 (PDB ID: 6V74). A comparative analysis of docking against 3 binding sites of PKM2 is provided in Table 2.

As for binding affinities, 15 compounds exhibit good binding energies (MolDock Score of >-145) to one or more of PKM2 binding sites. Three out of 15 compounds exhibit good binding affinities to all the 3 binding sites of PKM2. The top 3 common hits are Lupeollinoleate, Neochrome, and Maclurin 3-C-(6^″^-O-phydroxybenzoyl)*β*-Dglucoside. Docking interaction patterns of the top three hit compounds against FBP binding site of PKM2 are presented in Figure 4. These compounds possess good theoretical binding affinity with the target protein by mainly forming hydrogen bond and Van der Waals forces. Docking complexes of the best three *M. indica*-derived compounds against AA and PEP binding sites of PKM2 are presented in Figures 5 and 6, respectively.

The summary of enzymatic assay-based screening and virtual screening against PKM2 is provided in Figure 7.

## 4. Discussion

Targeting tumor metabolism has emerged as a novel and selective strategy for cancer therapy. A major metabolic difference associated with cancer is alteration in glucose metabolism. PK, a key enzyme that determines glycolytic activity, plays a critical role in cancer development [17]. Cancer cells express the specific M2 isoform (PKM2), and multiple evidences demonstrate that PKM2 expression support divergent biosynthetic and energetic requirements of cells in tumors. Unlike cancer cells, most of the normal tissues express another isoform of PK (PKM1). As PKM2 provides selective growth advantages to cancer cells over its counterpart PKM1, thus, targeting PKM2 provides an excellent opportunity for cancer therapies and drug development [18].

RETRACTED

PKM2 silencing has been known to induce apoptosis in cancer cells by recent studies [19]. PKM2 has also been reported to be highly expressed in various TNBC cell lines which provide further rationale for targeting PKM2 as novel anti-TNBC therapy [7].

Given that PKM2 inhibition has no effects on normal human breast tissues, PKM2 could serve as an ideal therapeutic target for TNBC [7] and it is of immense interest to identify and develop its inhibitors from natural products.

After screening of plant extract library, we identified *M. indica* (leaf, bark, and seed coat) extracts as PKM2 activity inhibitors at a final dose of 90 *μ*g/ml. Previous studies indicate that natural products from *Alkanna tinctoria* and *Arnebia* spp. exhibit PKM2 inhibitory activity. The extracts from these potentially active plants contain bioactive naphthoquinone compounds like alkannin, shikonin, and their derivatives [20]. Another natural compound lapachol has been found to be the potential inhibitor of PKM2 activity, leading to reduced ATP production and inhibition of cellular proliferation in human melanoma cells [4]. Berberine, isolated from *Coptis* and *Hydrastis canadensis*, has also been found to inhibit PKM2 activity leading to antitumor activity in HCT116 and HeLa cells [21]. Apigenin, naturally found in parsley, oranges, and onions, has been reported to block tumor glycolysis via inhibiting PKM2 expression and activity which in turn induced anticancer effects in colon cancer cells [22], indicating that blocking PKM2 activity by natural products has potential to halt the proliferation in tumor cells.

*M. indica* (leaf, bark, and seed coat) extracts also found to possess anticancer potential against highly aggressive breast cancer, TNBC. Our results are found to be concordant with the previous studies reporting anticancer potential of *M. indica* L. extracts against liver, colon, cervical, and gastric cancers [23, 24]. In order to explore new natural scaffolds from *M. indica* and provide further opportunities for anticancer drug discovery, we have screened *M. indica*-derived compounds against PKM2 by molecular docking. *In silico* based screening has identified several modulators of PKM2 which have potential to bind with AA, FBP, and PEP binding site of PKM2. From identified hits, neoxanthin has been previously known to inhibit chemically induced carcinogenesis in an *in vivo* hamster model [25]. Another hit compound, neochrome, is metabolite of neoxanthin which possess antiproliferative potential against prostate cancer cells [26]. Thus, the comparison of our results with existing literature suggests the potential of neoxanthin and neochrome as anticancer agents which might be due to PKM2 inhibition.

RETRACTED

## 5. Conclusions

Conclusively, enzymatic assay-based screening was performed to identify the plant extracts having potential to inhibit PKM2. This screen identified *M. indica* extracts as potential inhibitors of PKM2. Further *in silico* based screening identified various PKM2 modulators from *M. indica*. Although *M. indica* (bark and seed) extracts have been previously reported to possess significant anticancer potential, however, the underlying mechanism remains enigmatic. To the best of our knowledge, this is the first study which discloses that the *M. indica* exerts anticancer effects against TNBC via PKM2 inhibition. This study laid the foundation for further investigations to validate the efficacy of identified compounds against PKM2 via enzymatic activity assay. Although these findings suggest *M. indica* extracts as PKM2 inhibitors, however, further research is also recommended to test their potential in *in vivo* studies.

## Figures and Tables

**Figure 1:** Protein expression, purification, and establishment of enzymatic activity assay. (a) Double enzyme digestion for checking of insert. (b) Purity check of the purified recombinant PKM2 protein. (c) Principle of PKM2 enzymatic activity assay. (d) Optimization of substrate concentration (PEP) for PKM2 enzymatic assay.

**Figure 2:** Relative (%) PKM2 activity by varying concentration of *M. indica* leaf, bark, and seed coat extracts.

**Figure 3:** Dose-dependent growth inhibitions of MDA-MB231 cells by *M. indica* bark, leaf, and seed extracts.

**Figure 4:** Docking complexes of the best three *M. indica* compounds within the FBP binding site of PKM2.

**Figure 5:** Representation of docking complexes of top three ligands into the AA binding site of PKM2.

**Figure 6:** Interaction of hit compounds with amino acid residues at the PEP binding site of PKM2.

**Figure 7:** Summary of target protein-based screening of plant extract library and *in silico* based screening of *M. indica*-derived compounds against PKM2.

**Table 1:** Preliminary screening of crude plant extract library for the identification of PKM2 inhibitors.

Sr. no.	Plant name	Family	Common name	Part used	Extract no.	PKM2 activity
1	*Cyamopsis tetragonoloba* (L.) Taub	Fabaceae	Guar gum	Seeds	1	−
2	*Calotropis procera* (Aiton) Dryand.	Apocynaceae	Sodom apple	Leaves	2	−
3	*Azadirachta indica* A. Juss.	Meliaceae	Indian lilac	Leaves	3	−
4	*Ageratum conyzoides* L.	Asteraceae	Goat weed	Whole plant	4	−
5	*Dalbergia sissoo* sensu Miq.	Fabaceae	Indian rosewood	Seeds	5	−
				Bark	6	−
6	*Albizia lebbeck* (L.) Benth.	Fabaceae	Lebbeck	Flowers	7	−
				Seeds	8	−
				Seed coat	9	−
				Leaves	10	+
7	*Momordica charantia* L.	Cucurbitaceae	Bitter melon	Vegetable	11	−
				Seeds	12	−
8	*Oxalis corniculata* L.	Oxalidaceae	Creeping woodsorrel	Whole plant	13	−
9	*Cassia fistula* L.	Fabaceae	Golden shower	Leaves	14	+
				Fruit	15	+
10	*Aloe barbadensis* Mill.	Asphodelaceae	Aloe vera	Whole plant	16	−
11	*Nerium oleander* L.	Apocynaceae	Oleander	Leaves	17	−
12	*Chenopodium album* L.	Amaranthaceae	Lamb's quarters	Whole plant	18	−
13	*Bombax ceiba* L.	Malvaceae	Cotton tree	Leaves	19	−
				Bark	20	++
14	*Cicer arietinum* L.	Fabaceae	Chickpea (white)	Seed	21	−
			Chick pea (black)	Seed	22	−
15	*Smilax china* L.	Smilacaceae	China root	Roots	23	−
16	*Eucalyptus camaldulensis* Dehnh.	Myrtaceae	Himalayan poplar	Bark	24	−
17	*Helianthus annuus* L.	Asteraceae	Sun flower	Seeds	25	−
18	*Artemisia absinthium* L.	Asteraceae	Common wormwood	Whole plant	26	+
19	*Litchi chinensis* Sonn.	Sapindaceae	Lychee	Seeds	27	−
				Bark	28	+
				Leaves	29	−
20	*Lawsonia inermis*	Lythraceae	Henna	Leaves	30	−
21	*Cyperus esculentus* L.	Cyperaceae	Water grass	Flowers	31	−
22	*Fagonia arabica* L.	Zygophyllaceae	Dhamasa	Whole plant	32	−
23	*Cucumis melo agrestis* Naudin	Cucurbitaceae	Wild melon	Leaves	33	−
				Stem	34	−
24	*Asphodelus tenuifolius* Cav.	Asphodelaceae	Wild onion	Whole plant	35	−
25	*Solanum nigrum* L.	Solanaceae	Black nightshade	Whole plant	36	−
26	*Mangifera indica* L.	Anacardiaceae	Mango	Fruit pulp	37	−
				Peel	38	−
				Bark	39	++
				Seed coat	40	++
				Leaves	41	++
27	*Trachyspermum ammi* (L.) Sprague	Apiaceae	Carom seeds	Seeds	42	−
28	*Ferula assa-foetida* L.	Umbelliferae	Heng	Resin	43	−
29	*Linum usitatissimum* L.	Linaceae	Flax seeds	Seeds	44	−
30	*Citrullus colocynthis* (L.) Schrad.	Cucurbitaceae	Desert bitter gourd	Fruit	45	−
31	*Trigonella foenum-graecum* L.	Fabaceae	Fenugreek	Seeds	46	−
32	*Punica granatum* L.	Lythraceae	Pomegranate	Fruit peel	47	−
				Seeds	48	−
33	*Acacia farnesiana* (L.) Willd.	Fabaceae	Thorn Mimosa	Seeds	49	−
34	*Coriandrum sativum* L.	Apiaceae	Coriander	Seeds	50	−
35	*Citrus maxima* (Burm.) Merr.	Rutaceae	Chinese grapefruit	Peel	51	−

RETRACTED

**Table 2:** Docking results of *M. indica*-derived compounds against different binding site of PKM2.

Compound name	FBP binding site		AA binding site		PEP binding site	
	MolDock Score	HBond	MolDock Score	HBond	MolDock Score	HBond
Lupeollinoleate	-195.03	-5.03	-158.135	-3.14911	-183.99	-5.44131
Neochrome	-163.73	-5.31	-163.218	-8.04216	-142.153	-4.8914
Tetra-O-galloylglucose	-157.20	-35.16	-193.459	-19.630	-130.615	-28.8154
Neoxanthin	-155.84	-5.00	-120.848	-4.71265	-153.167	-6.0305
Luteoxanthin	-148.74	-3.55	-143.937	-3.779	-134.169	-4.93468
Gamma-tocopherol	-146.94	-4.99	-138.311	-6.75642	-108.115	-4.37926
*β*-Carotene	-145.99	0.00	-146.335	0	-129.354	0
Zeaxanthin	-144.59	-2.52	-144.795	0	-134.096	-0.798168
Beta-tocopherol	-142.54	-5.61	-125.241	-3.94614	-133.965	-1.92741
Mangiferic acid	-141.59	-4.79	-126.118	-1.45213	-129.938	-2.10352
Maclurin 3-C-(6^″^-O-phydroxybenzoyl)*β*-Dglucoside	-141.11	-19.75	-185.504	-30.6823	-152.56	-29.1472
Cryptoxanthin	-139.99	0.00	-144.965	0	-146.105	-1.91568
3-Methoxy-2-(4′-methyl benzoyl)-chromone	-132.76	-9.86	-120.813	-4.29266	-102.599	-4.55386
Apigenin 7-glucoside	-131.70	-27.05	-112.568	-6.71948	-100.576	-15.5694
Violaxanthin	-128.58	-0.49	-119.488	-1.81432	-88.3268	-7.52592
9-cis-Lutein (lutein)	-127.19	-2.35	-136.35	-2.5	-142.497	0
Mangiferin-6′-O-gallate	-125.08	-23.94	-112.949	-22.8972	-103.519	-26.8348
Rhamnetin	-124.29	-20.48	-110.02	-13.7748	-115.109	-10.6913
Epicatechin gallate	-123.03	-15.86	-103.822	-14.8456	-91.3209	-21.6137
Quercetin	-123.02	-22.78	-110.428	-12.0814	-110.252	-11.1415
Maclurin	-121.60	-15.94	-111.415	-8.34809	-97.7143	-14.8418
Rhamnetin hexoside	-120.91	-15.68	-110.437	-10.9705	-77.4519	-13.2685
Quercetin 3-O-rhamnoside	-120.80	-12.94	-115.172	-11.7603	-87.4993	-21.5166
Ellagic acid	-117.80	-15.43	-87.435	-9.7998	-72.6948	-11.7498
Ferulic acid	-117.17	-18.61	-105.778	-7.67901	-89.8163	-1.45049
Kaempferol	-115.78	-13.68	-107.609	-11.5349	-85.1987	-4.76716
*γ*-Sitosterol	-115.47	0.00	-90.502	-2.36888	-60.0014	-0.4356
Apigenin	-114.03	-14.49	-102.655	-10.3857	-108.222	-11.2041
*α*-Farnesene	-109.14	0.00	-102.741	0	-104.068	0
Syringic acid	-107.06	-10.80	-97.8327	-5.54318	-82.3703	-8.07737
Catechin	-106.29	-16.81	-85.0592	-8.07189	-72.7696	-15.0371
Quercetin carboxylic acid	-106.26	-31.53	-147.825	-24.6151	-131.161	-18.669
Caffeic acid	-104.79	-16.96	-100.104	-8.29169	-84.0058	-7.97793
Alpha-tocopherol	-104.68	0.00	-93.3105	0	-109.057	-2.5
Quercetin carboxylic acid	-101.33	-17.05	-78.7161	-16.5643	-61.109	-21.0371
Elemicin	-100.85	-1.95	-98.532	-3.63297	-80.2126	0
Campesterol	-100.76	0.00	-92.344	-2.5	-67.2379	-4.41775
p-Coumaric acid	-100.03	-15.79	-106.985	-5.2956	-88.197	-11.3534
Stigmasterol	-98.57	-2.50	-109.341	-3.17755	-79.599	-7.28574
Ethyl gallate	-98.32	-15.70	-91.6331	-11.2495	-95.4522	-17.0114
Mangiferin	-95.60	-23.65	-62.7887	-12.7153	-46.4801	-9.84916
Penta-O-gallose-glucose	-93.54	-16.92	-140.348	-27.0176		
*α*-Cubebene	-93.39	0.00	-73.0146	0	-80.0748	-1.51948
Methyleugenol	-92.76	0.00	-81.484	-1.37587	-78.2553	0
Gallic acid	-91.66	-18.00	-97.1975	-10.3128	-72.1728	-11.0514
Humulene	-90.71	0.00	-61.618	0	-63.6181	0
Theogallin	-90.31	-18.97	-68.6305	-19.8959	-79.8986	-21.7922
Iriflophenone-di-O-galloyl glucoside	-89.47	-20.70	-93.1958	-11.7291	-69.9375	-17.7076
Methyl gallate	-89.00	-15.10	-79.6082	-9.30537	-88.5411	-15.4398
*α*-Guaiene	-88.71	0.00	-69.7068	0	-63.3114	0
Dehydroascorbic acid	-87.17	-20.05	-75.4451	-15.0859	-77.1176	-13.908
Ascorbic acid	-87.12	-22.48	-84.9714	-13.4832	-70.4795	-16.0717
29-Hydroxymangiferonicacid	-86.95	-5.10	-80.1064	-5.24553	-50.0767	-12.6962
*α*-Sitosterol	-85.59	-0.78	-90.9633	-4.75248	-77.87	-3.2075
Protocatechuic acid	-85.59	-16.13	-93.325	-7.21244	-70.7263	-9.9475
Cinnamic acid	-84.63	-7.22	-93.9566	-4.03022	-76.26	-5.39073
Estragole	-83.21	-4.99	-79.9985	-0.38853	-80.1188	-0.484549
*δ*-Elemene	-81.71	0.00	-66.5298	0	-61.4269	0
Terpinyl acetate	-81.53	-2.98	-74.9132	-0.97568	-70.4852	-2.99327
Vanillin	-80.14	-11.30	-77.7569	-4.78744	-74.7439	-4.53428
Myrcene	-80.04	0.00	-77.3758	0	-86.4075	0
Linalool	-79.69	-5.37	-81.62	-5	-85.1614	-2.3688
Ocimene	-79.26	0.00	-81.2441	0	-84.1246	0
Mangiferonic acid	-79.13	-5.19	-77.262	-6.28465	-64.86	-8.29727
24-Methylenecycloartane-3*β*,26-diol	-78.22	-1.43	-78.4328	-2.93017	-64.4235	-9.29597
*β*-Bulnesene	-77.62	0.00	-72.542	0	-63.9464	0
Sabinene	-75.23	0.00	-81.1319	0	-73.5542	0
*β*-Elemene	-73.68	0.00	-61.4113	0	-54.1936	0
*γ*-Terpinene	-73.18	0.00	-74.3906	0	-65.0567	0
*γ*-Cadinene	-72.33	0.00	-48.6785	0	-50.5432	0
Dammarenediol II	-72.02	-5.26	-50.9481	-3.73546	-44.3381	-6.83216
Cycloartane-3,24,25-triol	-71.53	-8.76	-56.5961	-6.19957	-42.7277	-7.07424
Benzoic acid	-70.68	-7.57	-88.9444	-4.49511	-58.6953	-1.48964
Cymene	-70.26	0.00	-75.1263	0	-69.7851	0
*α*-Terpinolene	-68.95	0.00	-74.3397	0	-66.6623	0
*α*-Pinene	-67.71	0.00	-72.5574	0	-63.4011	0
Mangiferolate B	-66.67	-5.45	-54.2368	-4.18714	-49.3208	-3.97387
Limonene	-65.77	0.00	-72.9592	0	-63.0344	0
Pyrogallol	-64.60	-13.01	-68.5738	-9.57125	-63.477	-9.66407
Car3-ene	-63.20	0.00	-69.2717	0	-61.3925	0
Shikimic acid	-62.90	-15.54	-67.0134	-11.6281	-46.58	-12.5796
Resinol	-59.58	-9.91	-69.0014	-5	-60.3014	-7.5
*β*-Pinene	-59.12	0.00	-68.3213	0	-55.6667	0
Cycloartan-3*β*-30-diol cycloartan-3b	-59.10	-4.89	-70.9584	-7.08208	-33.8611	-1.92964
Camphene	-55.20	0.00	-66.3445	0	-52.2991	0
Eucalyptol	-53.56	-0.20	-63.9989	-2.39085	-48.9044	-0.155108
Quercetin pentoside	-47.75	-24.01	-77.8756	-11.9264	-87.2484	-29.9426
Manglupenone	-39.78	-5.75	-35.8728	-2.83316	-18.4948	-5
*β*-Sitosterol	-34.08	-0.99	-57.562	-3.78085	-43.5471	-4.42292
Lupeol	-33.19	-1.47	-32.275	-1.97739	-15.5679	-2.5
*β*-Amyrin	-28.02	-1.95	-28.957	-2.20045	-21.9474	0
Taraxerol	-27.67	0.00	-30.1279	-4.35048	-10.9574	-2.19296
Friedelin	-23.99	-4.34	-23.99	-4.34	-11.5989	-4.47101
*α*-Amyrin	-13.41	-1.86	-21.125	-0.17742	-8.75428	-1.11693

RETRACTED

## Data Availability

The data used to support the findings of this study are included within the article.
